# Functional analyses of microRNA-326 in breast cancer development

**DOI:** 10.1042/BSR20190787

**Published:** 2019-07-29

**Authors:** Ye Du, Lishengnan Shen, Wei Zhang, Rongbo Ding, Qian Li, Simin Li, Haipeng Zhang

**Affiliations:** 1 Department of Breast Surgery, The First Hospital of Jilin University, Changchun 130021, Jilin, P.R. China; 2 Department of Cosmetology Plastic Surgery the First Hospital of Jilin University, Changchun 130021, Jilin, P.R. China; 3 Department of Gynecology, the First Hospital of Jilin University, Changchun 130021, Jilin, P.R. China

**Keywords:** Breast cancer, invasion, miR-326, proliferation, SOX12

## Abstract

MicroRNA-326 (miR-326) was reported to be dysregulated and involved in the progression of multiple cancers. However, the clinical significance, biological role and underlying mechanism of miR-326 in the carcinogenesis of breast cancer are still unclear. In the present study, we showed that miR-326 was down-regulated in human breast cancer tissues and cell lines. Our results also revealed that miR-326 overexpression significantly suppressed breast cancer cell proliferation, migration and invasion, and induced cell cycle arrest at G_1_/G_0_ phase. Furthermore, Sex determining region Y-box (SOX) protein 12 (SOX12), a known oncogene, was identified as a direct target of miR-326 by luciferase reporter assay. Moreover, miR-326 expression was inversely correlated with *SOX12* mRNA expression levels in human breast cancer specimens. Overexpression of SOX12 partially rescued the inhibitory effect on cell proliferation, migration and invasion in breast cancer cells caused by miR-326 overexpression. These findings suggested that miR-326 might play a suppressive role in breast cancer, at least in part, by targeting SOX12, rendering miR-326 a promising therapeutic target for breast cancer.

## Introduction

Breast cancer is one of the most common malignant malignancies in women worldwide [1]. Despite considerable improvements in therapeutic strategies for breast cancer including multi-agent chemotherapy, surgery and radiotherapy, the 5-year survival rate of breast cancer has not improved significantly due to tumor metastasis and recurrence [2,3]. Therefore, it is urgently needed to understand the molecular mechanisms involved in development and progression of breast cancer for identifying novel and effective diagnosis markers and therapeutic targets.

MicroRNAs (miRNAs) are a class of short (19–25 nucleotide in length) and noncoding small RNA molecules that can result in translational repression and gene silencing by binding to the 3′-untranslated regions (3′-UTRs) of target genes [4]. Growing evidence has demonstrated the vital function of miRNAs in multiple biological processes, including proliferation, apoptosis, cycle arrest, differentiation, metabolism and metastasis [5]. Dysregulation of miRNAs have been revealed to be involved in initiation and development of various cancers [6,7]. Number of miRNAs was identified to be involved in progression of breast cancer, suggesting that miRNAs can serve as diagnosis marker and therapy agent [8–10].

MicroRNA-326 (miR-326) was reported to be down-regulated and function as tumor suppressor in multiple cancers, including lung cancer [11], hepatocellular carcinoma [12], prostatic carcinoma [13], gastric cancer [14], osteosarcoma [15], glioblastoma [16] and nasopharyngeal carcinoma [17]. However, the expression pattern, possible functions and underlying mechanisms of miR-326 are yet to be described in breast cancer.

Sex determining region Y-box protein (SOX) 12 (SOX12), an important member of the SOX family, was reported to play crucial roles in cardiac, neuronal and mesenchymal development processes [18]. Several studies reported that SOX12 is up-regulated and contribute to initiation and progression of several cancers, including gastric cancer [19], colorectal cancer [20], hepatocellular carcinoma [21] and lung cancer [22]. Recently a study showed that SOX12 expression was up-regulated in breast cancer tissues, and knockdown of SOX12 inhibited breast cancer proliferation, migration and invasion *in vitro*, and suppressed tumor growth *in vivo* [23], suggesting that SOX12 play an oncogenic role in breast cancer. However, the underlying causes of aberrant SOX12 expression in breast cancer are unclear.

In the present study, we found that miR-326 expression was significantly decreased in breast cancer tissues and cells. We also found that miR-326 overexpression led to impaired proliferation, migration and invasion of breast cancer cells by partially targeting SOX12, suggesting that miR-326 play a tumor suppressive role in breast cancer.

## Materials and methods

### Patient samples

Breast cancer specimens and adjacent normal tissues were collected from 48 patients who underwent surgery in the First Hospital of Jilin University (Changchun, China) from January 2014 to December 2016. None of the patients received radiotherapy, chemotherapy or any other treatment before and after operation. The patients included 20 cases at clinical stage I, 18 cases at stage II, 8 cases at stage III and 2 cases at stage IV. Breast tumors and normal tissue specimens excised surgically from patients were immediately snap-frozen in liquid nitrogen for miR-326 and SOX12 assays. The present study has been carried out in accordance with the World Medical Association Declaration of Helsinki, and that all subjects provided written informed consent. The use of tissue samples were approved by the ethical committees of the First Hospital of Jilin University.

### Cell culture and transfection

Human normal breast epithelial cell line MCF-10A and four breast cancer cell lines (MCF-7, MDA-MB-231, MDA-MB-468 and BT-474) were bought from the American Type Culture Collection (ATCC, Rockville, MD). All cells were grown in RPMI-1640 (Gibco, CA, U.S.A.) supplemented with 10% fetal bovine serum (FBS; Gibco) and incubated at 37°C in a 5% CO_2_ incubator.

The miR-326 mimics (miR-326, 5′-CCUCUGGGCCCUUCCUCCAG-3′) and the appropriate negative control mimic (miR-NC, 5′-UUCUCGAACGUGUCACGUUUU-3′) were designed and synthesized from Guangzhou RiboBio Co., Ltd (Guangzhou, China). The SOX12-overexpression vector (pCDNA3.1-SOX12) was a kind gift from Dr. Wei Zhang (Jilin University). MCF-7 cells were transiently transfected with mimics or the overexpression vector using Lipofectamine® 2000 (Invitrogen; Thermo Fisher Scientific, Inc) based on manufacturer’s protocol. Transfection efficiency was examined in every experiment at 48 h post-transfection.

### Reverse transcription-quantitative polymerase chain reaction analysis

Total RNA was extracted from cultured cells and tissues using TRIzol® reagent (Invitrogen; Thermo Fisher Scientific, Inc.) according to the manufacturer’s instructions. The expression levels of miR-326 were examined using the TaqMan MicroRNA assay Kit (Thermo Fisher Scientific, Inc.) under an ABI 7900 real-time PCR system (Thermo Fisher Scientific, Inc.) following the manufacturer’s instructions. For the detection of *SOX12* mRNA, complementary DNAs (cDNAs) were synthesized from RNA templates by using a PrimeScript First-Strand cDNA synthesis kit (Takara Biotechnology Co., Ltd., Dalian China) according to the manufacturer’s protocol. The cDNAs were then amplified using SYBR Premix ExTaq II (TaKaRa Bio Technology Co., Ltd) in an ABI 7900 real-time PCR system. The primers used in the present study are listed in Table 1. Relative quantification of the target genes was performed using the 2^−ΔΔ*C*^_t_ method by ABI software [24]. U6 and GAPDH were assessed as endogenous controls for miR-326 and SOX12, respectively.

**Table 1:** The primers used in the present study

Target gene	Primer (5′–3′)
*U6*	F-TCCGATCGTGAAGCGTTC
	R-GTGCAGGGTCCGAGGT
*miR-326*	F-CCTCTGGGCCCTTCCTCCAG
	R-GCTGTCAACGATACGCTACCTA
*SOX12*	F-AAGGGCGTCGTGGTTCCAACTC
	R-AGCATTGCCGTCCTGGGTGTAG
*GAPDH*	F-AAGGTGAAGGTCGGAGTCAA
	R-AATGAAGGGGTCATTGATGG
*WT-SOX12*	F-CCGCTCGAGTCAGGAACAAACGGTCCCAGAGT
	R-ATAAGAATGCGGCCGCACTCTGGGACCGTTTGTTCCTGA
*Mut-SOX12*	F-CCGCTCGAGTCAGGAACAAACGGTGGGTCTCA
	R-ATAAGAATGCGGCCGCTGAGACCCACCGTTTGTTCCTGA

Abbreviations: F, forward; GAPDH, glyceraldehyde-3-phosphate dehydrogenase; MT, mutant-type; R, reverse; WT, wild-type.

### Cell proliferation

A total of 5 × 10^3^ transfected cells were seeded in 96-well plates in RPMI-1640 medium supplemented with 10% FBS for 24–72 h. Then cell proliferation was examined with a Cell Counting Kit-8 (CCK-8; Dojindo Laboratories, Kumamoto, Japan) according to the manufacturer’s protocol. The optical density (OD) was read at 450 nm using a Benchmark Plus microplate spectrometer (Bio-Rad Laboratories, Hercules, CA, U.S.A.). The experiment was repeated three times.

### Cell cycle arrest detection

MCF-7 cells were harvested at 48 h post-transfection. Then cells were and fixed in 70% ethanol at −20°C overnight. Subsequently, transfected cells were stained with propidium iodide (PI, Beijing Solarbio Science and Technology Co., Ltd. Beijing, China) in the presence of RNaseA for 15 min. Finally, cell cycle arrest was determined using flow cytometer (BDLSR II, BD Biosciences, Franklin Lakes, NJ, U.S.A.). Cell cycle distribution was analyzed using CellQuest 3.0 software (BD Biosciences). The experiment was repeated three times.

### Wound healing assay

Cell migration ability was measured by a wound healing assay *in vitro*. Briefly, 2 × 10^4^ transfected cells were seeded on to six-well plates, and grown to 100% confluence. Subsequently, an artificial homogeneous wound was scratched into the monolayer using a sterile plastic micropipette tip and incubated in fresh medium free of FBS for 24 h. Finally, the wound width was measured by the ImageJ software (NIH, Bethesda, MD, U.S.A.). Wound closure was imaged at 0 and 24 h after scratching using an inverted microscope (Olympus Corporation, Tokyo, Japan). The experiment was repeated three times.

### Transwell invasion assay

Transwell insert chambers (Corning Inc., Corning, NY, U.S.A.) were applied to evaluate cell invasion ability. Briefly, 1 × 10^5^ transfected cells were seeded into upper chamber precoated with Matrigel (BD, Franklin Lakes, NJ, U.S.A.) in serum-free medium, and medium containing with 10% FBS was added to the lower chamber as a chemoattractant. After incubation for 48 h at 37°C, cells that had invaded the lower chamber surface were fixed with 70% ethanol and stained with 1% Crystal Violet for 30 min at 37°C. The invading cells were imaged and counted at five selected random fields using an inverted microscope (Olympus Corporation). The experiment was repeated three times.

### Bioinformatics, miRNA-target identification and luciferase assay

A predication software TargetScan (http://www.targetscan.org/vert_71/) was used to predict potential targets of miR-326. The relationship between miR-326 and SOX12 in breast cancer cells was determined by using a luciferase reporter assay. The wild-type (WT) putative binding site in the 3′-UTR of SOX12 or its mutant-type (MT) was amplified and inserted into the psiCHECK2 luciferase reporter vector (Promega Corporation, Madison, WI, U.S.A.), and designated as WT-SOX12 and MT-SOX12, respectively. The primes used in the present study were listed in Table 1. For the luciferase assay, MCF-7 cells were grown to 70–80% confluence in 24-well plates and co-transfected with an miR-326 mimic or miR-NC (at the final concentrations of 50 nM) and WT-SOX12 or MT-SOX12 reporter plasmids (200 ng) using Lipofectamine 2000 (Invitrogen) following the manufacturer’s protocol. Luciferase activity was examined using a dual-luciferase reporter assay (Promega Corporation) at 48 h post-transfection. *Renilla* luciferase activity was normalized against that of firefly luciferase. The experiment was repeated three times.

### Western blot assay

Total proteins were collected from tissues and cultured cells using RIPA buffer (Solarbio, Beijing, China). The concentrations of proteins were measured using bicinchoninic acid (BCA) assay kit (Beyotime, Biotechnology, Shanghai, China). The proteins were separated using 10% sodium dodecyl sulfate/polyacrylamide gel electrophoresis (SDS/PAGE) and electro-transferred on to polyvinylidene fluoride (PVDF) membrane (Reno, Hangzhou, China) in a semi-dry blotting apparatus (Bio-Rad, Hercules, California). After blocking with TBST-soluble 5% dried skimmed milk at room temperature for 2 h, the membranes were respectively bound to the mouse monoclonal anti-human SOX12 antibody (1:1000; Abcam, Cambridge, MA, U.S.A.) or mouse monoclonal anti-human GAPDH (1:5000; Santa Cruz Biotechnology Inc, CA, U.S.A.) at 4°C overnight. Then membrane was bound to the corresponding secondary antibodies (Rabbit anti-mouse IgG, 1:6000; Abcam) at 37°C for 1 h. The blots were assessed using an enhanced chemiluminescence reagent (ECL, GE Healthcare, Chicaogo, IL, U.S.A.).

### Statistical analysis

All data were expressed as the mean ± standard deviation (SD) from three independent repeats of the experiments. SPSS v. 19.0 (IBM Corp., Armonk, NY, U.S.A.) was used for statistical analyses. Student’s *t* test was employed for comparisons between two groups. One-way analysis of variance was used to estimate the significant differences among multiple groups. Pearson’s correlation analysis was used to analyze correlation with miR-326 and SOX12 in breast cancer tissues. In all the cases, differences were considered significant when *P*-values were less than 0.05.

## Results

### miR-326 expression was down-regulated in breast cancer tissues and cell lines

The expression levels of miR-326 in 48 paired tissue samples including breast cancer tissues and corresponding adjacent normal tissues were initially examined. The results of reverse transcription quantiative polymerase chain reaction (qRT-PCR) revealed that the expression levels of miR-326 were abnormally down-regulated in breast cancer tissues compared with adjacent normal tissues (Figure 1A). Moreover, the expression of miR-326 expression was lower in clinical stage III–IV patients with breast cancer than that in clinical stage I–II patients (Figure 1B). Meanwhile, the expressions of miR-326 in breast cancer cells (MCF-7, MDA-MB-231, MDA-MB-468 and BT-474) and normal breast epithelial cell line MCF-10A were also measured by qRT-PCR. As compared with human normal breast epithelial cell line (MCF-10A), the expression of miR-326 was significantly decreased in breast cancer cell lines (Figure 1C). Notably, the expression of miR-326 was more evident in MCF-7 cells than in other three breast cancer cells. Hence, MCF-7 cells were selected for subsequently all experiments.

**Figure 1:** miR-326 expression was down-regulated in breast cancer tissues and cell lines (**A**) qRT-PCR analysis of miR-326 expression in 48 paired tissue samples including breast cancer tissues and corresponding adjacent normal tissues. (**B**) qRT-PCR analysis of miR-326 expression in 38 clinical stage I–II breast cancer patients and 10 clinical stage III–IV breast cancer patients. (**C**) qRT-PCR analysis of miR-326 expression in four breast cancer cell lines (MCF-7, MDA-MB-231, MDA-MB-468 and BT-474) and human normal breast epithelial cell line (MCF-10A). Data are presented as the means ± SD (n=3). **P<0.01.

### miR-326 inhibited breast cancer cell proliferation and induced cell cycle at G_1_/G_0_ phase

To investigate whether miR-326 played a key role in the progression of breast cancer, MCF-7 cells were transfected with miR-326 mimics or miR-NC. As shown in Figure 2A, transfection with miR-326 mimics resulted in a remarkable increase in the expression of miR-326 in MCF-7 cells compared with transfection with miR-NC, suggesting that transfection efficiency was successful. Subsequently, the effects of miR-326 on cell viability and cell cycle were investigated. CCK-8 assay showed that overexpression of miR-326 significantly decreased cell viability of MCF-7 cells at 48–96 h (Figure 2B). Since cell proliferation was closely associated with cell cycle arrest, thus, we investigated the effect of miR-326 on cell cycle arrest by flow cytometry assay. Our results revealed that transfection miR-326 mimics in MCF-7 cells significantly increased cell cycle arrest at G_1_/G_0_ stage and decreased cell cycle arrest at S stage compared with cells transfected with miR-NC (Figure 2C). These results suggested that miR-326 inhibited breast cancer cell proliferation by regulating cell cycle arrest at G_1_/G_0_ stage.

**Figure 2:** miR-326 inhibited breast cancer cell proliferation and induced cell cycle at G_1_/G_0_ phase (**A**) The expression levels of miR-326 were measured in MCF-7 cells transfected with miR-326 mimics or miR-NC by qRT-PCR. (**B**) Cell proliferation was measured in MCF-7 cells transfected with miR-326 mimics or miR-NC by CCK-8 assay. (**C**) Cell cycle distribution was examined in MCF-7 cells transfected with miR-326 mimics or miR-NC by flow cytometry. Data are presented as the means ± SD (n=3). *P<0.05; **P<0.01.

### miR-326 inhibited breast cancer cell migration and invasion

Next, we sought to explore the influence of miR-326 on migration and invasion of MCF-7 cells by wound healing assay and transwell invasion assay, respectively. The results revealed that overexpression of miR-326 markedly reduced the migration and invasion abilities of MCF-7 cells (Figure 3A,B).

**Figure 3:** miR-326 inhibited breast cancer cell migration and invasion (**A**) Cell migration was examined in MCF-7 cells transfected with miR-326 mimics or miR-NC using a wound-healing assay. (**B**) Cell invasion was determined in MCF-7 cells transfected with miR-326 mimic or miR-NC by a Transwell invasion assay. Data are presented as the means ± SD (n=3). **P<0.01.

### SOX12 was a direct target of miR-326 in breast cancer cells

Growing evidence suggested that miRNAs exert their function in cancer cells by regulating target gene [5]. To explore underlying mechanism that miR-326 inhibited proliferation and metastasis of MCF-7 cells, we used TargetScan software to search for candidate targets of miR-326, finding that the SOX12 3′-UTR matched the miR-326 seed sequence (Figure 4A). To further verify whether SOX12 was a direct target of miR-326 in breast cancer cells, a luciferase-reporter assay was performed in MCF-7 cells, revealing that overexpression of miR-326 clearly inhibited the luciferase activity of the WT-SOX12 3′-UTR, not but that of MT-SOX12 3′-UTR activity (Figure 4B). Moreover, overexpression of miR-326 in MCF-7 cells markedly reduced SOX12 mRNA and protein levels (Figure 4C,D). Additionally, we also examined *SOX12* mRNA expression in breast cancer tissues and cell lines, and found that *SOX12* expression was up-regulated in breast cancer tissues and cell lines compared with adjacent normal tissues and cell line (Figure 4E,F). *SOX12* expression was higher in clinical stage III–IV patients than that in clinical stage I–II patients (Figure 4G). Pearson’s correlation analysis revealed that *SOX12* mRNA levels were inversely correlated with miR-326 expression levels in breast tissues (*r* = −0.412; *P*=0.008; Figure 4H). These results suggested that SOX12 was a target of miR-326 in breast cancer cells.

**Figure 4:** SOX12 was a direct target of miR-326 in breast cancer cells (**A**) miR-326 and its putative binding sequence in the SOX12 3′-UTR. A mutated binding site was generated in the miR-326 seed region. (**B**) Luciferase activity was determined in MCF-7 cells co-transfected with miR-326 mimics or miR-NC, and luciferase reporter vector containing WT-SOX12 or MT-SOX12. (**C,D**) SOX12 expression on mRNA and protein levels was examined in MCF-7 cells transfected with miR-326 mimics or miR-NC by qRT-PCR. (**E**) The mRNA expression of *SOX12* was examined in 48 paired tissue samples including breast cancer tissues and corresponding adjacent normal tissues. (**F**) The mRNA expression of *SOX12* was examined in four breast cancer cell lines (MCF-7, MDA-MB-231, MDA-MB-468 and BT-474) and human normal breast epithelial cell line (MCF-10A).(**G**) The mRNA expression of *SOX12* was determined in 38 clinical stage I–II breast cancer patients and 10 clinical stage III–IV breast cancer patients. (**H**) A significant inverse correlation between the *SOX12* mRNA levels and miR-326 was observed in breast cancer tissues. Data are presented as the means ± SD (n=3). *P<0.01.

### SOX12 overexpression partially rescued cells from the biological effects of miR-326 induction in breast cancer cells

To investigate whether miR-326 exerted its biological functions by regulating SOX12, the present study restored SOX12 expression by transfecting a SOX12-overexpression plasmid (pCDNA3.1-SOX12) into miR-326-overexpressing MCF-7 cells (Figure 5A,B). In addition, our results also revealed that restoration of SOX12 partially abrogated the effect of miR-326-overexpressing MCF-7 cells proliferation, cycle arrest, migration and invasion (Figure 5C–F).

**Figure 5:** SOX12 overexpression partially rescued cells from the biological effects of miR-326 induction in breast cancer cells (**A,B**) SOX12 expression on mRNA and protein levels was measured in MCF-7 cells after transfection with miR-326 mimics with (or without) the SOX12*-*overexpression vector (pCDNA3.1-SOX12) or miR-NC. (**C**–**F**) Cell proliferation, cycle arrest, migration and invasion were determined in MCF-7 cells after transfection with miR-326 mimic with (or without) pCDNA3.1-SOX12 or miR-NC. Data are presented as the means ± SD (n=3). *P<0.05; **P<0.01.

## Discussion

Accumulating evidence has suggested that dysfunction of miRNAs played crucial roles in the initiation and progression of breast cancer via regulating their targets [8–10]. For example, Qin and Liu [25] reported that miRNA-99a-5p suppressed breast cancer progression and cell cycle pathway through targeting CDC25A. Zhu et al. [26] showed that miR-196b-5p inhibited cell growth and metastasis in breast cancer through down-regulating collagen type I α 1 chain (COL1A1). Guo et al. [27] demonstrated that miR-508-3p inhibited cell invasion and epithelial–mesenchymal transition by targeting ZEB1 in breast cancer. The major finding of the current study was that miR-326 inhibited proliferation and invasion of breast cancer cells through targeting SOX12, revealing a novel epigenetic mechanism of how miR-326 played a tumor suppressive role in breast cancer.

Growing evidence has shown that miR-326 functioned as a tumor suppressor in multiple types of malignant tumors [11–17]. Although a study showed that miR-326 implicate in chemotherapy resistance of breast cancer through regulating expression of multidrug resistance-associated protein 1 [28], its functional role and underlying mechanism in breast cancer remained largely unknown. In the current study, we identified for the first time that the tumor suppressor role of miR-326 in breast cancer by a series of experiments. We found that the expression of miR-326 was dramatically reduced in breast cancer tissues and cell lines, and its expression was closely negatively associated with clinical stage of patients with breast cancer. Functional experiments demonstrated that miR-326 overexpression significantly inhibited breast cancer cell proliferation, migration and invasion, and induced cell cycle arrest at G_1_/G_0_ phase. These results suggested that miR-326 played a suppressive role in breast cancer progression.

It was well known that miRNAs exerted biological role by regulating their target genes [5]. Thus, to investigate the underlying mechanisms by which miR-326 exerts its anti-cancer effects on breast cancer, it is necessary to identify its targets. TargetScan software was used to identify target of miR-326. Among targets, SOX12, a member of the Sox (SRY-related HMG-box) family of transcription factors, was selected as a candidate target for further investigation based on its biological function [29]. Recently a study showed that SOX12 expression was up-regulated in breast cancer tissues, and that SOX12 played an oncogenic role in promoting growth, migration and invasion of breast cancer cells [23]. Here, through luciferase-reporter assay, qRT-PCR and Western blot analysis, SOX12 was further identified as a direct target of miR-326 in breast cancer cells. Furthermore, our results showed that miR-326 expression was inversely correlated with *SOX12* mRNA levels in breast cancer tissues. Importantly, our results also revealed that restoration of SOX12 expression partially abrogated the functional effect of miR-326 on breast cancer cell proliferation, cycle arrest, migration and invasion. These data provided reliable evidence suggesting that miR-326 exerted an inhibitory effect on breast cancer progression, at least in part, by targeting SOX12.

Some limitations exist in the present study. First, enough breast cancer samples are needed to further investigate clinical significance of miR-326. Second, *in vivo* experiments need be performed to clarify miR-326 functional role in breast cancer. Third, miRNAs could target multiple mRNAs, thus, the detailed regulatory mechanisms of miR-326 on breast cancer progression should be further explored in future research.

In conclusion, our results demonstrated that miR-326 was down-regulated in breast cancer tissue samples and cell lines. miR-326 functioned as a tumor suppressor in breast cancer by inhibiting proliferation, invasion and migration via partially targeting SOX12. Therefore, miR-326 might serve as a therapy target for breast cancer.

## Abbreviations

CCK-8: Cell Counting Kit-8
CDC25A: Cell division cycle 25A
cDNA: complementary DNA
FBS: fetal bovine serum
HMG: Human menopausal gonadotropin
miR-326: microRNA-326
MT: mutant-type
qRT-PCR: Reverse transcription quantitative polymerase chain reaction
RIPA: Radio immunoprecipitation assay
RPM1640: Roswell park memorial institute 1640
SOX12: Sex determining region Y-box protein 12
WT: wild-type
ZEB2: Zinc finger E-box-binding homebox2
3′-UTR: 3′-untranslated region
